# The Role of Osthole on TGF-*β*-Induced Lung Epithelium Apoptosis Injury and Epithelial-Mesenchymal Transition-Mediated Airway Remodeling in Pediatric Asthma

**DOI:** 10.1155/2022/7099097

**Published:** 2022-03-24

**Authors:** Jinghai Tang, Jilong Liu, Xuehua Zhang

**Affiliations:** ^1^Department of Pediatrics, Maternal and Child Health Hospital of Shandong Province, Jinan, Shandong 250014, China; ^2^Department of Common Pediatric, Shandong Cao County People's Hospital, Heze, Shandong 250014, China

## Abstract

Osthole, a coumarin compound derived from Fructus Cnidii, exerts anti-inflammatory effects in an asthma model. But the effect of osthole on epithelial injury and epithelial-mesenchymal transition (EMT) in asthma remains unclear. 16HBE cells were incubated with TGF-*β*1 with or without osthole in vitro. Ovalbumin (OVA)-induced asthmatic mouse model was established in vivo. Cell counting kit-8 was carried out to evaluate the viability of 16HBE cells. The impact of osthole on TGF-*β*1-evoked cell apoptosis and EMT process was measured by flow cytometry based on Annexin V-FITC/PI staining, transwell assay, immunofluorescence, and Western blot. The regulatory role of osthole in TGF-*β*1/Smad and p38, ERK1/2, and JNK MAPK signaling was detected via Western blot. Osthole treatment significantly suppressed TGF-*β*1-induced 16HBE cell apoptosis, verified by a reduced percentage of apoptotic cells, decreased expression of proapoptotic proteins (cleaved-caspase3 and Bax), and enhanced antiapoptotic factor (Bcl-2) expression. In addition, the promotive impact of TGF-*β*1 on the migration of 16HBE cells was reversed by osthole, accompanied by elevated E-cadherin expression and reduced Snail and N-cadherin expression. The activation of the Smad2/3 and MAPKs pathway evoked by TGF-*β*1 was inhibited by osthole in 16HBE cells. We also found that osthole mitigated airway epithelium injury and subepithelial fibrosis in OVA-challenged asthmatic mice in vivo. Osthole could mitigate TGF-*β*1-induced epithelial cell injury and EMT process by suppressing the activation of MAPK and Smad2/3 pathways separately. Our present study showed a new insight into understanding the underlying mechanism of osthole injury on epithelium injury and subepithelial fibrosis in airway remodeling. Asthma, epithelial injury, epithelial-mesenchymal transition, and airway remodeling are the effects of osthole on airway remodeling.

## 1. Introduction

Bronchial asthma in children is a common chronic respiratory disease, which poses a serious threat to children's health. Airway remodeling, as an important pathologic characteristic, is involved in the pathogenesis of bronchial asthma. A series of studies have shown that the airway remodeling process exists in the pathogenesis of paediatric asthma [1, 2].

The airway epithelial barrier is critical to defense against the stimulation of allergens and its integrity depends on tight junctions and adherens junctions, orchestrating the relationship between airway inflammation and airway remodeling [3]. In paediatric asthma, continual epithelial injury and repair could elicit the onset of airway remodeling [4–7]. When repeatedly stimulated by allergens and pathogens, airway epithelium undergoes shedding caused by apoptotic injury, contributing to the loss of integrity of the epithelial barrier [8, 9]. While, repeated repair mediated by epithelial-mesenchymal transition (EMT) is associated with the pathogenesis of subepithelial fibrosis in airway remodeling [4]. Therefore, directly targeting airway epithelium is considered as a novel therapeutic strategy for airway remodeling in childhood asthma.

Osthole, one of the most important coumarin compounds isolated from the ripe fruit, is derived from the Umbelliferae plant *Cnidium monnieri* (L.) Cuss. Increasing studies have shown that osthole has biological functions such as antitumor, liver protection, anti-inflammation, neuroprotection, and antiapoptosis[10, 11]. For example, osthole can suppress apoptosis of cardiomyocytes and inflammation in monocrotaline-induced right ventricle remodeling [12]. Kordulewska et al. showed that osthole reduces histine-induced increased COX-2 expression in peripheral blood mononuclear cells (PMBC) with or without symptoms of allergies/asthma in autistic children, thereby enhancing anti-inflammatory effects [13]. Osthole has been found to play an anti-inflammatory role in asthma models [14, 15]. Osthole can inhibit the EMT process of a variety of diseases, including lung cancer and renal fibrosis [16, 17]. However, the effect and underlying mechanism of osthole on the apoptosis injury and EMT process of epithelial cells in asthma remain unclear.

During the pathogenesis of airway remodeling, TGF-*β*1, as an important growth factor, evokes epithelial apoptosis and EMT, leading to epithelial shedding and subepithelial fibrosis in asthma [18]. TGF-*β*1-mediated activation of the downstream pathway can be divided into two types: the Smad pathway and the non-Smad pathway, of which the non-Smad pathway mainly includes PI3K/AKT and MAPKs pathways. TGF-*β*1 can trigger human bronchial epithelial cell apoptosis through ERK/p38/JNK MAPK signaling pathways [19]. Pu et al. demonstrated that the apoptosis process of TGF-*β*1-stimulated bronchial epithelial BEAS-2B cells is associated with the MAPK pathway, while the process of EMT is related to the TGF-*β*/Smad and MAPK pathway [20]. Previous reports demonstrated that osthole can regulate the EMT process of prostate cancer through the TGF-*β*/Akt/MAPK pathways [21, 22]. Here, we wonder whether TGF-*β*1-activated Smad and MAPK pathways are implicated in the regulatory function and underlying mechanism of osthole in bronchial epithelial cells.

Taken together, the present study was conducted with the purpose of exploring the regulatory function and relative mechanism of osthole in airway epithelial apoptosis and EMT-evoked defective epithelium repair in airway remodeling of asthma in children.

## 2. Methods

### 2.1. Cell Culture and Treatment

Human bronchial epithelial 16HBE cells were obtained from the Cell Bank of the Chinese Academy of Sciences (Shanghai, China). Cells were cultured in RPMI-1640 with 10% fetal bovine serum (FBS, GIBCO, USA) and 100 U/ml penicillin and 100 ug/ml streptomycin under an atmosphere of 5% CO_2_ at 37°C. After starvation in serum-free medium for 6–8 h and pretreatment with TGF-*β*1 (10 ng/ml, R&D system, USA) for 24 h, cells were cotreated with or without osthole (MedChemExpress, China) for another 24 h. DMSO was used to dissolve osthole, and osthole was stored as a stock solution at concentration of 1 mM, followed by diluting with culture medium for the subsequent assay.

### 2.2. Cell Viability Assay

The viability of 16HBE cells with incubation of osthole at a series of concentrations including 0, 2.5, 5, 10, 20, and 40 *μ*M for 24 h was evaluated by the cell counting kit-8 (Beyotime, China). A total of 2500 cells in 100 *μ*L complete medium (RPMI-1640 + 10% FBS) were added into wells in a 96-well plate. CCK-8 reagent (10 *μ*L) was diluted with RPMI-1640 at a ratio of 1 : 10, and then, 100 *μ*L working solution was added into wells. After incubating for 2 h, the absorbance value at 450 nm was measured with a microplate reader.

### 2.3. Cell Apoptosis Assay

Flow cytometry based on Annexin V-FITC/PI staining was carried out to detect the ratio of apoptotic cells. Cells (3 × 105/well) were incubated in 6-well plates for 48 h. Cells and culture medium in each well were harvested and followed by the detection in accordance with manufacturer's instruction.

### 2.4. Western Blotting

Tissues and cells were lysed with RIPA lysis buffer to extract total protein. The protein quantification kit (Sigma-Aldrich, USA) was employed to quantify the protein concentration. The same amount of proteins were isolated using 8–10% SDS-PAGE and subsequently blotted onto PVDF (Millipore, USA). After blocking, the membranes were incubated with the primary antibody overnight at 4°C. The primary antibodies from Cell Signaling Technology and Santa Cruz included E-cadherin (1 : 700 diluted), N-cadherin (1 : 600 diluted), Snail (1 : 1100 diluted), Bcl-2 (1 : 900 diluted), Bax (1 : 800 diluted), cleaved-caspase3 (1 : 700 diluted), Smad2/3 (1 : 1100 diluted), p-Smad2 (1 : 1100 diluted), p-Smad3 (1 : 1200 diluted), ERK (1 : 1200 diluted), p-ERK (1 : 1200 diluted), p38 (1 : 1200 diluted), p-p38 (1 : 1200 diluted), JNK (1 : 1200 diluted), p-JNK (1 : 1200 diluted), TGF-*β*1 (1 : 1500 diluted), and *β*-actin (1 : 2000 diluted). After washing, membranes were exposed to specific secondary antibodies (1 : 5000, ZSGB-BIO, China) for 60 min at room temperature. Then, band intensity was detected with an ECL kit (Millipore, USA) and analyzed using Image J software.

### 2.5. Quantitative RT-PCR

A TRIzol reagent (Beyotime, China) was used to extract total RNA in accordance with the instructions provided. EasyScript® First-Strand cDNA Synthesis SuperMix (TransGen, China) was employed for reverse-transcription of RNA. The expression quantity of mRNA was evaluated by qPCR using the TransStart® Green qPCR kit (TransGen, China) on the Roche LightCycler 96 (Roche, Germany). Primers in this analysis are given in Table 1. The 2^−△△Ct^ method was performed to analyze the fold change of genes, and GAPDH was considered as a reference.

### 2.6. Transwell Assay

Transwell chambers (Corning, USA) with an 8 *μ*m pore size was used to measure cell migratory ability. 16HBE cells were resuspended in 100 *μ*l RPMI-1640 without serum and plated in the upper chamber, while 550 *μ*l 10% serum-RPMI-1640 containing TGF-*β*1 (10 ng/mL) and osthole (OST, 10 *μ*M) was supplemented in the lower chamber. After incubation for 24 h, cells across the membrane of the upper chamber were fixed and then stained with 0.1% crystal violet solution. A cotton swab was used to wipe up the cells below the upper chamber gently. Five fields were observed and randomly counted using an inverted microscope.

### 2.7. Immunofluorescence Staining

After fixed with 95% ethanol and blocked with 1% BSA, cells were incubated using rabbit anti-E-cadherin (1 : 150 diluted) antibody and rabbit anti-N-cadherin (1 : 150 diluted) antibody overnight at 4°C, respectively. Then, goat anti-rabbit IgG/PE labeled secondary antibody was added for cell incubation for 1 h in the dark. Afterwards, cells were stained with DAPI for nucleus staining. Images were observed and captured with a fluorescence microscope.

### 2.8. Asthmatic Mouse Model

Female young BALB/c mice (*n* = 18), aged 5-week-old, were fed adaptively for one week in standard experimental animal center before experiments. 10 *μ*g OVA (Sigma-Aldrich, USA) and 1 mg aluminium hydroxide adjuvant in 200 *μ*l sterile PBS were injected intraperitoneally on days 1, 7, and 14 for two weeks to sensitize mice in the OVA-challenged group. Mice with intraperitoneal injection using PBS were involved in the control group. Then, the mice were aerosolized with 1% OVA in PBS solution for 30 min once a day for15–21 days, and the mice in the OVA-challenged group were intraperitoneally injected with saline and OST (50 mg/kg) 2 h before OVA inhalation. All mice were euthanized on day 22. The lung tissues were collected for protein detection by Western blotting and histopathological examination by staining with H&E and Masson.

### 2.9. H&E Staining

4% formalin-fixed and paraffin-embedded specimens were sectioned into 5 *μ*m thick sections and then deparaffinized, followed by rehydrated with a series of graded alcohols. Slices were stained with hematoxylin, followed by hydrochloric acid alcohol differentiation and then were stained with eosin solution. After mounted on neutral mounting medium (Sigma-Aldrich, USA), the histopathologic change of lung bronchial tissues was visualized under a light microscope.

### 2.10. Masson Staining

Histological examination of lung bronchial tissues' fibrosis was evaluated by Masson's trichrome staining. Paraffin-embedded specimens were sectioned into 5 *μ*m thick sections and then deparaffinized and gradient rehydrated. Weigert hematoxylin solution was used to stain slices for 6 min. After washing adequately, slices were stained with Ponceau fuchsin acid solution for 6 min, immersed with 2% glacial acetic acid solution for 60 s, and with 1% phosphomolybdic acid water solution for 4 min for differentiation. Then, without washing, aniline blue solution was used to stain for 5 min, and 0.2% glacial acetic acid solution was employed to soak the slices for 1 min. After that, slices were dehydrated with graded alcohol and vitrificated by xylene. Finally, neutral resin was used to mount the slices.

### 2.11. Data Analysis

All results were represented as mean ± SD and analyzed statistically using Graphpad prism (Graphpad Software, USA). Student's *t*-test and one-way ANOVA followed by Bonferroni's post-hoc test were applied to compare differences between two groups or among multiple groups separately. *P* < 0.05 was deemed as statistical significance.

## 3. Results

### 3.1. Osthole Suppressed TGF-*β*1-Induced Bronchial Epithelial Cells 16HBE Apoptosis

Figure 1(a) shows the molecular structure of osthole. The cytotoxic effect of osthole at different doses on 16HBE cells was measured by the cell counting kit-8. As shown in Figure 1(b), osthole at the low concentrations (2.5, 5, and 10 *μ*M) had no significant cytotoxic effect on 16 HBE cells, while 20 and 40 *μ*M of osthole resulted in a sharp reduction in cell viability compared with the group without osthole treatment (*P* < 0.001), indicating that cell viability was inhibited with the increased concentration of osthole. Subsequently, we detected the effect of osthole at various concentrations (0, 2.5, 5, and 10 *μ*M) on TGF-*β*1-evoked apoptosis of 16HBE cells. As described previously [23], TGF-*β*1 (10 ng/ml) was used to prestimulate cells for 24 h, followed by treatment in combination with or without osthole for a further 24 h. TGF-*β*1 treatment dramatically enhanced 16HBE cell apoptosis, which was suppressed by osthole in a concentration-dependent manner in comparison with the control group (Figure 1(c)). Next, we detected cell apoptosis-related protein levels by immunoblotting. TGF-*β*1 markedly upregulated the protein level of Bax and cleaved-caspase3 while impairing Bcl-2 expression, which was dramatically attenuated by osthole treatment (Figure 1(d)). These results showed that osthole suppressed TGF-*β*1-induced 16HBE cell apoptosis. On consideration of the more significant suppression effect of 10 *μ*M of osthole on TGF-*β*1-induced 16HBE cell apoptosis, 10 *μ*M of osthole was used in the following experiments.

### 3.2. Osthole Inhibited Epithelial-Mesenchymal Transition of 16HBE Induced by TGF-*β*1

To explore the regulatory role of osthole in TGF-*β*1-evoked 16HBE cell migration, transwell assay was carried out. As shown in Figure 2(a), TGF-*β*1 significantly promoted the number of migrated 16HBE cells, while the effect was alleviated by the treatment of 10 *μ*M of osthole. We found that TGF-*β*1 induced a change of cell morphology. Compared with the control group, the typical epithelial oval morphology of 16HBE cells changed to spindle fibroblast-like morphology in the TGF-*β*1 + DMSO group, while in the TGF-*β*1+OST group, cells regained the epithelial morphology (Figure 2(b)). Next, we put focus on the suppression mechanism of osthole on 16HBE cell migration stimulated by TGF-*β*1; therefore, we detected the mRNA and protein levels of N-cadherin, Snail (mesenchymal marker), and E-cadherin (epithelial marker) using qRT-PCR and immunoblotting. Osthole treatment significantly reversed the promotive effect of TGF-*β*1 on N-cadherin and Snail expression and had an inhibitive effect on the expression of E-cadherin at both mRNA and protein levels (Figures 2(c) and 2(d)). The result of immunofluorescence assay showed that TGF-*β*1 stimulation caused a dramatic reduction of E-cadherin protein level and increased N-cadherin expression in 16HBE cells, while the above effects were effectively blocked by osthole treatment (Figures 2(e) and 2(f)). These results revealed that osthole treatment inhibited TGF-*β*1-stimulated EMT in 16HBE cells.

### 3.3. Osthole Suppressed 16HBE Cell Apoptosis and EMT via Regulating TGF-*β*1-Mediated Activation of MAPK and Smad Signaling Pathways

TGF-*β*1-mediated signaling pathways, such as Smad2/3, p38, ERK1/2, and JNK MAPK, play important roles in epithelium injury and the EMT process in asthma [24, 25]. Therefore, we first detected the related protein expression of the Smad2/3 and MAPKs pathway by Western blot to explore whether the regulatory mechanism of osthole treatment on cell apoptosis and EMT of 16HBE cells with TGF-*β*1 induction was associated with activation of the Smad2/3 and MAPKs pathway mediated by TGF-*β*1. Osthole treatment significantly reduced TGF-*β*1-elevated phosphorylation level of ERK1/2, p38, JNK, Smad2, and Smad3, thereby revealing the suppression impact of osthole on activation of the Smad2/3 and MAPKs pathway (Figures 3(a) and 3(b)). A recent study reported that TGF-*β*1 induced bronchial epithelial cell apoptosis via the MAPK signaling pathway [20]. Therefore, we detected the effect of MAPK inhibitors on 16HBE cell apoptosis induced by TGF-*β*1. We found that MAPK inhibitors (SP600125, SB203580, and PD98059) significantly suppressed the proportion of apoptotic cells evoked by TGF-*β*1 (Figure 3(c)). Next, the expression of Smad2 and Smad3 were successfully decreased by transfection of siRNA-Smad2 or siRNA-Smad3, respectively (Figure 3(d)). Based on the function of Smad2/3 signaling on EMT, we detected the protein levels of E-cadherin, N-cadherin, and Snail by immunoblotting. The result of Figure 3(d) demonstrated that E-cadherin expressed at a higher level, and the protein level of Snail and N-cadherin was lower in the TGF-*β*1+si-Smad2 group and TGF-*β*1+si-Smad3 group than in the TGF-*β*1+si-NC group. Then, the transwell assay was applied to evaluate the impact of Smad2/3 knockdown on TGF-*β*1-evoked cell migratory ability. Silencing of Smad2 or Smad3 inhibited TGF-*β*1-induced migrated cell number, respectively (Figure 3(e)). The above results demonstrated that osthole suppressed the activation of MAPK and TGF-*β*1/Smad2/3 signaling pathways and then inhibited TGF-*β*1-induced 16HBE cell apoptosis and EMT process.

### 3.4. Osthole Could Alleviate the Epithelium Injury and Subepithelial Fibrosis in Asthmatic Mice

We assessed the effect of osthole on airway remodeling in the OVA-exposed mouse in vivo. H&E staining was carried out to observe the histopathologic change of lung tissue. In OVA-exposed mice, there were significant infiltrated inflammatory cells around bronchus compared with the control group, while treatment with osthole alleviated the inflammatory cell infiltration (Figure 4(a)). Increasing reports have shown that the pathogenesis of subepithelial fibrosis in airway remodeling is attributed to TGF-*β*1-induced EMT [26, 27]. Masson's staining demonstrated that OVA challenge in the OVA + saline group induced enhanced collagen deposition and increased collagen fiber compared with the control group; when treated with osthole, there was a significant decrease in depth of collagen deposition (Figure 4(b)). Then, we evaluated the expression of EMT-related proteins in lung tissues by Western blot. We found that osthole treatment reversed the downregulated E-cadherin and upregulated Snail and N-cadherin of lung tissues in OVA-exposed mice (Figure 4(c)). Furthermore, osthole treatment attenuated OVA-induced increased level of TGF-*β*1 and elevated phosphorylated levels of Smad2 and Smad3 in lung tissues (Figure 4(d)). Next, we investigated the regulatory function of osthole on the epithelial injury of lung tissues. We found that OVA challenge enhanced the protein levels of Bax, cleaved-caspase3, and caused impaired Bcl-2 expression; injection of osthole suppressed the effect of OVA on the above protein (Figure 4(e)). To further investigate the mechanism of osthole in epithelial damage in OVA-induced mice, we detected the MAPK signaling pathway in lung tissues by Western blot. In the OVA + saline group, there were prominent activation of ERK1/2, p38, and JNK in lung tissues in comparison with the control group, while with the administration of osthole, the phosphorylation levels of ERK, p38, and JNK were decreased (Figure 4(f)). These results demonstrated that osthole treatment could alleviate EMT-induced subepithelial fibrosis and cell apoptosis-elicited airway epithelium injury via TGF-*β*1/Smad2/3 and MAPKs pathways separately in young mice exposed to OVA.

## 4. Discussion

Airway remodeling, the typical hallmark of bronchial asthma, could result in restricted airflow, airway stenosis, and airway hyperresponsiveness. Increasing evidences revealed that airway remodeling plays an important role in the pathogenesis of peadiatric asthma [28, 29]. Treatment against the development of airway remodeling becomes a new therapy target for asthma in children. In the present study, we investigate the effective therapeutic role of osthole for the first time, as a natural antihistamine alternative. Its roles in the pathogenesis of airway remodelling, particularly on airway epithelial apoptosis and EMT-induced subepithelial fibrosis, were investigated in vitro and in vivo.

Epithelium damage, the pathologic feature characteristic of adult asthma, is present even in children with asthma [30]. Defective epithelium injury repair mediated by the EMT process can contribute to airway fibrosis. Therefore, it is necessary to inhibit excessive apoptosis of airway epithelial cells and epithelium injury repair during treatment of airway remodeling. A previous report showed that azithromycin can suppress airway epithelial cell apoptosis to mitigate airway remodeling in asthma model rats [25]. Huangqi-Fangfeng abates the EMT process to relieve airway remodeling in asthma mice exposed to house dust mite (HDM) [31]. In our present study, we established the airway remodeling model in vitro by treating bronchial epithelial cell 16HBE with TGF-*β*1. Our results demonstrated that TGF-*β*1 stimulated 16HBE cell apoptosis and proapoptotic protein cleaved-caspase3 and Bax levels were upregulated, and antiapoptotic protein level of Bcl-2 was reduced, which were consistent with the previous reports [20, 25, 23]. With the treatment of osthole, TGF-*β*1-induced 16HBE cell apoptosis was inhibited, indicating that osthole could relieve bronchial epithelium apoptosis injury. In addition, accompanied by osthole treatment, the migrated cell number was reduced in TGF-*β*1-stimulated 16HBE cells. Osthole caused increased E-cadherin but impaired N-cadherin and Snail in 16HBE cells evoked by TGF-*β*1. More importantly, intraperitoneal injection of osthole could significantly alleviate the airway inflammation and collagen deposition, and this was consistent with the previous study [15]. Moreover, we found that osthole can also suppress the cell apoptosis and EMT process in OVA-induced asthma mice. These results demonstrated the treatment effect of osthole in airway remodeling of asthma.

TGF-*β*1, as a critical growth factor, can elicit the pathogenesis of airway epithelium injury and EMT-induced airway fibrosis in asthma. The activation of Smad2/3 and MAPKs signaling was the important downstream of the TGF-*β*1-mediated pathway and can result in tissue fibrosis and inflammation in various disease [32, 33]. Osthole was reported to function by blocking the TGF-*β*1/MAPK pathway [21, 34]. In this study, we showed that osthole could inhibit the activation of TGF-*β*1/Smad2/3 and ERK1/2, p38, JNK MAPK signaling, thus contributing to the suppression of EMT and cell apoptosis in airway epithelium, respectively, in the experimental asthma model in vitro and in vivo. However, it remains to be verified whether the inactivation of Smad2/3 takes part in epithelial cell apoptosis.

In conclusion, our present study demonstrated that osthole could suppress cell apoptosis and EMT process in bronchial epithelium via MAPK and TGF-*β*1/smad2/3 signaling pathways, thereby alleviating airway epithelium injury and EMT-induced subepithelial fibrosis during the pathogenesis of airway remodeling in paediatric asthma. This present study revealed the effect of osthole on bronchial epithelium in airway remodeling and the adjuvant therapeutic potential of osthole for bronchial asthma in children.

## Figures and Tables

**Figure 1:** The impact of osthole on TGF-*β*1-induced cell apoptosis in 16HBE cells. 16HBE cells pretreated with TGF-*β*1 (10 ng/ml) for 24 h and then cotreated in combination with osthole (2.5, 5, and 10 *μ*M) or not for further 24 h. (a) Molecular structure of osthole. (b) Cell viability of 16HBE cells treated with osthole at the various doses for 24 h detected by the CCK-8 kit. (c) The apoptosis of 16HBE cells detected by flow cytometry. (d) The protein level of Bcl-2, Bax, and cleaved-caspase3 detected by Western blot. ^∗∗^*P* < 0.01, ^∗∗∗^*P* < 0.001, no significance versus the indicated group.

**Figure 2:** The effect of osthole on TGF-*β*1-induced epithelial-mesenchymal transition in 16HBE cells. 16HBE cells were treated with TGF-*β*1 (10 ng/ml) with or without osthole (10 *μ*M) for 24 h. (a) The migrative ability of 16HBE cells determined by transwell assay (*n* = 5). (b) Changes in cell morphology observed via inverted microscopy (x100). (c) The mRNA levels of epithelial markers (E-cadherin) and mesenchymal marker (N-cadherin and Snail) in 16HBE cells detected by qRT-PCR. (d) Western blot performed to measure the protein levels of E-cadherin, N-cadherin, and Snail in 16HBE cells. (e) The expression of E-cadherin (red) evaluated by immunofluorescence staining, and nucleus was stained with DAPI (blue) (x200). (f) N-cadherin (red) expression evaluated by IF staining, and nucleus was stained with DAPI (blue) (x200). ^∗∗^*P* < 0.01, ^∗∗∗^*P* < 0.001 versus the indicated group.

**Figure 3:** Osthole inhibited MAPK and TGF-*β*/Smad pathways in TGF-*β*1-induced 16 HBE cells. (a) The total levels and phosphorylated levels of Erk1/2, p38, and JNK of the MAPK signaling pathway determined by Western blot. (b) The phosphorylation levels of Smad2, Smad3, and total levels of Smad2/3 detected by Western blot. (c) The effect of MAPK inhibitor on TGF-*β*1-induced apoptosis in 16HBE cells detected by flow cytometry, SP600125: JNK inhibitor, SB203580: p38 inhibitor, and PD98059: Erk inhibitor. After transfected with the si-NC vector, or si-Smad2 vector, or si-Smad3 vector for 48 h, 16HBE cells were induced by TGF-*β*1. (d) Western blot performed to detect the expression of Smad2, Smad3, Snail, E-cadherin, and N-cadherin. (e) Transwell assay carried out to detect cell migration (*n* = 5). ^*∗*^*P* < 0.05, ^∗∗^*P* < 0.01, ^∗∗∗^*P* < 0.001, no significance versus the indicated group.

**Figure 4:** Osthole attenuated epithelial injury and EMT in OVA-exposed mice. (a) Histopathologic examination of lung bronchial tissues evaluated by hematoxylin and eosin staining (upper panel 200x and lower panel 400x). (b) Masson's staining performed to show the change in tissue fiber around the bronchus (400x). (c) The expression of E-cadherin, N-cadherin, and Snail in lung tissues detected by Western blot. (d) The expressions of TGF-*β*1, phosphorylated level of Smad2 and Smad3, and total Smad2/3 in lung tissues measured by Western blot. (e) The change in protein levels of Bax, Bcl-2, and cleaved-caspase3 in lung tissues examined by Western blot. (f) The phosphorylated level and total level of the MAPK signaling pathway detected by Western blot. ^*∗*^*P* < 0.05, ^∗∗^*P* < 0.01, ^∗∗∗^*P* < 0.001 versus the indicated group.

**Table 1:** Primers for real-time PCR.

	Gene forward primer (5′ to 3′)	Reverse primer (5′ to 3′)

E-cadherin	CGAGAGCTACACGTTCACGG	GGGTGTCGAGGGAAAAATAGG
N-cadherin	TGCGGTACAGTGTAACTGGG	GAAACCGGGCTATCTGCTCG
Snail	TCGGAAGCCTAACTACAGCGA	AGATGAGCATTGGCAGCGAG
GAPDH	GGAGCGAGATCCCTCCAAAAT	GGCTGTTGTCATACTTCTCATGG

## Data Availability

The datasets used to support the findings of this study are available from the corresponding author upon request.

## Abbreviation

OST: Osthole
TGF-*β*1: Transforming growth factor *β*1
OVA: Ovalbumin
CCK-8: Cell counting kit-8
MAPK: Mitogen-activated protein kinase
PI: Propidium iodide
DMSO: Dimethyl sulfoxide
PBS: Phosphate-buffered saline
PVDF: Polyvinylidene fluoride
SDS-PAGE: Sodium dodecyl sulfate-polyacrylamide gel electrophoresis
SD: Standard deviation
ANOVA: One-way analysis of variance
HDM: House dust mite
FBS: Fetal bovine serum.
